# lncRNA FGD5-AS1 and miR-130a Can Be Used for Prognosis Analysis of Patients with Chronic Periodontitis

**DOI:** 10.1155/2021/8544914

**Published:** 2021-12-10

**Authors:** Miao Yu, Chunyuan Chi

**Affiliations:** Department of Stomatology, Weifang People's Hospital, Weifang, 261000 Shandong Province, China

## Abstract

**Background:**

lncRNA and microRNA affect the occurrence and development of many diseases, so they are expected to become diagnostic or predictive indicators. But the relationship between lncRNA FGD5-AS1 and miR-130a and the prognosis of chronic periodontitis is still unclear. The purpose of this study is to explore the prognostic value of the two in chronic periodontitis.

**Objective:**

This study set out to investigate the prognostic value of lncRNA FGD5-AS1 and miR-130a in chronic periodontitis.

**Methods:**

Eighty-seven patients with chronic periodontitis who visited our hospital from March 2016 to August 2017 were collected as an observation group (OG), and 72 subjects with periodontal health who underwent physical examination at the same time were collected as a control group (CG). The FGD5-AS1 and miR-130a expression levels of subjects in the two groups were compared, and prognosis of 87 patients who were reviewed one year later was counted. The expression levels of patients with different prognoses were compared when they were admitted to our hospital. We drew the ROC curve and explored the prognostic value of FGD5-AS1 and miR-130a. The risk factors for adverse prognosis were analyzed through logistic regression.

**Results:**

FGD5-AS1 was lowly expressed in patients, while miR-130a was highly expressed. FGD5-AS1 and miR-130a had certain diagnostic and predictive value in chronic periodontitis and patient prognosis. The higher the periodontal pocket, the higher the attachment loss. Lower FGD5-AS1 and higher miR-130a levels were independent prognostic risk factors.

**Conclusion:**

lncRNA FGD5-AS1 is lowly expressed in patients with chronic periodontitis, while miR-130a is highly expressed. Both of them have certain diagnostic and prognostic value in chronic periodontitis and may be potential diagnostic and prognostic indicators.

## 1. Introduction

Periodontitis is the most common inflammatory disease in the world, which affects about 50% of adults and 60% of people over 65 years old. It is also an oral disease with extremely high morbidity in China [1, 2]. It is often caused by poor oral hygiene and bacterial infection. The release of inflammatory factors after its onset will destroy the balance of alveolar bone absorption and attachment, resulting in bone loss and gradual destruction of oral tissues [3]. Inflammation of chronic periodontitis has long duration. Soft tissue and hard tissue around teeth will be affected, which will often lead to tooth loss or dentition dysfunction in patients at the later stage of development [4]. Moreover, there are also some references showing that the risk of chronic periodontitis patients complicated with cardiovascular diseases, chronic respiratory diseases, cancer, and other diseases is dramatically higher than that of people without chronic periodontitis, so the treatment and control of chronic periodontitis become critical [5]. Prognosis of patients in the treatment of chronic periodontitis is a key point that we must consider, so that we can better adjust the treatment plan and support effective treatment decisions [6].

Long noncoding RNA (lncRNA) is a noncoding single-stranded RNA with a length of more than 200 nucleotides [7]. There are some lncRNA that affect the development of periodontitis, and their expression levels are dramatically different between patients and normal people [8]. lncRNA FGD5-AS1 is an lncRNA [9] discovered recently that can interfere with the development of periodontitis through the SOCS6/NF-KB pathway. However, it is still unclear whether FGD5-AS1 can be used for prognostic analysis of patients with chronic periodontitis.

The regulation process of lncRNA is often to bind mRNA by acting as a competitive endogenous RNA (ceRNA) so as to target and regulate the microRNA and target protein expression levels to affect the occurrence and development of diseases [10]. ceRNAs are transcripts as microRNA spongesthat regulate each other at the post-transcriptional level through competitivebinding with other microRNAs. ceRNAs has been found to include protein-codingmRNAs and non-coding RNA, in which non-coding RNA includes pseudogene transcripts,lncRNA, and circular RNA etc. The presence of ceRNAs affect the functional activity ofmicroRNAs. ceRNAsactivity can form a large-scale transcriptional regulatory network, which canexpand the functional genetic information in the human genome and play a rolein pathological conditions. MicroRNA is an endogenous noncoding RNA, which also participates in the development and regulation of some diseases [11, 12]. Venugopal et al. [13] found that the miR-125b, miR-100, and miR-21 expression levels in periodontitis patients were abnormal with normal people and affected periodontitis through the interaction of some signal pathways and cytokines. miR-130a is an inflammation-related microRNA; it has abnormal expression in patients with osteoarthritis and leukemia inflammation, so does periodontitis [14–16]. However, there is little research on the prognostic value of lncRNA FGD5-AS1 and miR-130a in chronic periodontitis.

Therefore, in this study, we hope to observe the FGD5-AS1 and miR-130a expression levels in different prognoses of chronic periodontitis to analyse their prognostic value and provide the basis and direction for clinical practice.

## 2. Methods

### 2.1. Patient Data

Eighty-seven patients with chronic periodontitis who visited our hospital from March 2016 to August 2017 were collected as an observation group (OG), including 39 males and 48 females with an average age of 48.1 ± 9.5 years and an age range of 31-64 years. Seventy-two subjects with periodontal health who underwent physical examination during the same period were also collected as a control group (CG), including 41 males and 31 females with an average age of 47.6 ± 8.5 years and an age range of 26-60 years. This study was conducted with the approval of the Medical Ethics Committee, and all patients were informed and signed an informed consent form.

### 2.2. Inclusion and Exclusion Criteria

Inclusion criteria were as follows: patients were diagnosed with chronic periodontitis by imaging [17], no anti-inflammatory drugs were used for nearly 3 months, their clinical data were complete, and the treatment and follow-up were coordinated.

Exclusion criteria were as follows: patients had implant or orthodontic appliance, patients took bactericide orally in the past 3 months, patients had less than 18 natural teeth in the full mouth, and patients were complicated with diabetes.

### 2.3. Detection Methods

Specimens of gingival crevicular fluid from all subjects were collected and stored into EP tubes at -80°C for later use. The collected samples were extracted with the EasyPure miRNA kit, and the purity, concentration, and integrity were tested by using ultraviolet spectrophotometer and agarose gel electrophoresis. Total RNA was reversely transcribed through the TransScript® miRNA RT Enzyme Mix and 2×TS miRNA Reaction Mix (Transgen Biotech Co., Ltd., Beijing, ER601-01, AT351-01), and the operation steps were strictly in accordance with the manufacturer's kit. Then, PCR amplification experiment was carried out under a PCR instrument (ABI, USA, 7500). A PCR reaction system was as follows: cDNA 1 *μ*L, upstream and downstream primers 0.4 *μ*L each, 2×TransTaq® Tip Green qPCR SuperMix 10 *μ*L, passive reference dye (50×) 0.4 *μ*L, and ddH_2_O supplemented to 20 *μ*L. PCR reaction conditions were as follows: predenaturation at 94°C for 30 s, denaturation at 94°C for 5 s, and annealing at 60°C for 30 s. The above three steps had 40 cycles in total. Each sample was provided with 3 repeated wells, and the experiment was carried out 3 times. In this study, FGD5-AS1 used GAPDH as an internal reference, miR-130a used U6 as an internal reference, and 2^−△△ct^ was employed to analyze the data. The left and right primers were provided by Sangon Biotech (Shanghai) Co., Ltd., and the primer sequence is shown in Table 1.

### 2.4. Outcome Measures

#### 2.4.1. Main Outcome Measures

The differences of lncRNA FGD5-AS1 and miR-130a expression levels in the OG and the CG were compared, and the prognosis of the patients one year after discharge was counted. The prognosis was good if PD < 4 mm reexamined after one year and poor if PD ≥ 4 mm. According to their prognosis, they were divided into the good prognosis group (GPG) and poor prognosis group (PPG), and their independent prognostic risk factors were analyzed by multivariate logistic regression.

#### 2.4.2. Secondary Outcome Measures

The diagnostic value and prognostic value of FGD5-AS1 and miR-130a in patients with chronic periodontitis were analyzed by the receiver operating characteristic (ROC) curve.

### 2.5. Statistical Analysis

The collected data were statistically analyzed via SPSS 20.0 (SPSS Co., Ltd., Chicago, USA). Their pictures were drawn by using GraphPad Prism 7 (GraphPad Software Co., Ltd., San Diego, USA). The counting data usage was expressed as *n* (%) and checked by *X*^2^. The measurement data were expressed as mean ± standard deviation (mean ± SD), and all those conformed to normal distribution. Comparison between the two groups was under the independent samples *t*-test. Multivariate analysis of prognosis was under the multivariate logistic regression test. *P* < 0.05 indicates statistically significant differences.

## 3. Results

### 3.1. Clinical Data

By comparing the clinical data of the OG and the CG, we found that there was no remarkable difference in gender, age, BMI, and history of smoking or alcoholism of subjects between the two groups, while there were remarkable differences in the number of teeth, gingival index, plaque index, sulcus bleeding index, pocket depth, and attachment loss (*P* < 0.05) (Table 2).

### 3.2. Expression Differences and Diagnosis ROC of lncRNA FGD5-AS1 and miR-130a in the Two Groups

By comparing the lncRNA FGD5-AS1 and miR-130a expression levels in both groups, we found that FGD5-AS1 (0.51 ± 0.28) in the OG was obviously lower than that in the CG (1.03 ± 0.45) (*t* = 8.899, *P* < 0.001) (*P* < 0.05), and miR-130a (1.58 ± 0.44) in the OG was obviously higher than that in the CG (1.01 ± 0.32) (*t* = 9.166, *P* < 0.001) (*P* < 0.05). The ROC curve for diagnosis of chronic periodontitis revealed that the area under the lncRNA FGD5-AS1 curve was 0.835 and the best specificity and sensitivity were 88.51% and 72.22%, respectively, when the cut-off point was 0.805; the area under the miR-130a curve was 0.851 and the best specificity and sensitivity were 80.46% and 77.78%, respectively, when the cut-off point was 1.227; and the area under the joint detection curve was 0.929 and the best specificity and sensitivity were 80.46% and 90.28%, respectively, when the cut-off point was 0.321 (Figure 1, Table 3).

### 3.3. Expression of lncRNA FGD5-AS1 and miR-130a in Different Prognosis Groups and Diagnosis of ROC

Prognosis of the patients in the OG reviewed after one year was collected. Sixty-four patients had good prognosis and 23 patients had poor prognosis. According to their prognosis, they were divided into GPG (*n* = 64) and PPG (*n* = 23). The FGD5-AS1 expression levels (0.59 ± 0.25) in the GPG were markedly higher than those in the PPG (0.28 ± 0.23) (*t* = 5.205, *P* < 0.001) (*P* < 0.05). The miR-130a expression levels (1.45 ± 0.41) in the GPG were dramatically lower than those in the PPG (1.93 ± 0.34) (*t* = 5.023, *P* < 0.001) (*P* < 0.05). The predicted prognosis ROC curve revealed that the area under the lncRNA FGD5-AS1 curve was 0.822 and the best specificity and sensitivity were 90.63% and 60.87%, respectively, when the cut-off point was 0.237; the area under the miR-130a curve was 0.819 and the best specificity and sensitivity were 73.44% and 82.61%, respectively, when the cut-off point was 1.686; and the area under the joint detection curve was 0.916 and the best specificity and sensitivity were 81.25% and 82.61%, respectively, when the cut-off point was 0.295 (Figure 2, Table 3).

### 3.4. Univariate Analysis

Through univariate analysis of the clinical data of the GPG and the PPG, it was found that there were statistical differences in the gingival index, plaque index, sulcus bleeding index, pocket depth, attachment loss, FGD5-AS1, and miR-130a between the two groups (*P* < 0.05), while there were no statistical differences in gender, age, BMI, history of smoking, history of alcoholism, and number of teeth (*P* > 0.05) (Table 4).

### 3.5. Multivariate Analysis of Prognosis

We included the indicators with differences in univariate analysis into the evaluation (the evaluation table is shown in Table 5). Then, we chose to proceed with LR to perform multivariate logistic regression analysis. The results revealed that the gingival index, plaque index, and sulcus bleeding index were not independent risk factors for patients' prognosis, while periodontal pocket, attachment loss, FGD5-AS1, miR-130a, miR-17-5p, and miR-130a were independent risk factors for poor prognosis of patients (Table 6).

## 4. Discussion

Many evidences display that microRNA and lncRNA play a role in the occurrence and development of diseases, and the same regulatory mechanism exists in periodontosis [18–20]. Lian et al. [21] found that miR-335-5p could promote osteoblast activity and reduce periodontal bone destruction and inflammation in periodontitis, so as to prevent periodontitis and bone loss. Han et al. [22] discovered that lncRNA TUG1 could reduce inflammation caused by lipopolysaccharide and regulate cell proliferation and apoptosis of periodontal ligament cells.

In this research, we found that the FGD5-AS1 expression in periodontitis patients was remarkably lower than that in healthy people, while the miR-130a expression was remarkably higher than that in healthy people, suggesting that FGD5-AS1 and miR-130a expression levels were probably altered in patients. The ROC curve analysis found that the area under the FGD5-AS1 and miR-130a curve presented with considerable specificity and sensitivity, respectively, and the sensitivity of combined detection was better than that of single detection of two indexes. Additionally, we found that the FGD5-AS1 expression levels in patients with good prognosis were remarkably higher than those in patients with poor prognosis, while the miR-130a expression levels were remarkably lower than those in patients with poor prognosis; this indicated that the FGD5-AS1 and miR-130a expression levels were tied to the prognosis of periodontitis patients.

We then explored the independent risk factors for poor prognosis of patients with chronic periodontitis and found that the higher the periodontal pockets, the higher the loss of attachment; lower FGD5-AS1 and higher miR-130a levels were independent risk factors for their prognosis. In previous studies, age, bone height, and periodontal pocket were mentioned as prognostic factors of patients [23, 24], while our study first found that FGD5-AS1 and miR-130a were also independent prognostic factors of chronic periodontitis. Hence, in the future, we can predict the prognosis of patients through the levels of two indicators, so as to implement the corresponding treatment plans.

Nevertheless, there are still some limitations in this study. In the first place, the study did not consider the treatment plan of patients, so it was not clear whether different treatment plans would have different effects on the FGD5-AS1 and miR-130a expression levels, and whether there would be differences in their expression levels in patients with different efficacies had not been explored. In the second place, we did not study the specific mechanism of FGD5-AS1 and miR-130a regulating chronic periodontitis, and we did not predict the target gene and target protein mediated by the two. Finally, we were still not clear whether there was a certain relationship between FGD5-AS1 and miR-130a. Hence, we hope to increase the corresponding basic experiments in the later stage to explore the specific impact mechanism of FGD5-AS1 and miR-130a and their interrelation.

To summarize, lncRNA FGD5-AS1 is lowly expressed in patients with chronic periodontitis while miR-130a is highly expressed. Both of them have certain diagnostic and prognostic value in chronic periodontitis and may be potential diagnostic and prognostic indicators.

## Figures and Tables

**Figure 1:** Expression differences and diagnosis ROC curve of lncRNA FGD5-AS1 and miR-130a in the OG and CG. (a) FGD5-AS1 expression levels in the OG were dramatically lower than those in the CG (*t* = 8.899, *P* < 0.001). (b) miR-130a expression levels in the OG were dramatically higher than those in the CG (*t* = 9.166, *P* < 0.001). (c) ROC curve of lncRNA FGD5-AS1 and miR-130a in diagnosing chronic periodontitis. ∗∗∗ indicates *P* < 0.001.

**Figure 2:** Expression differences and prognosis ROC curve of FGD5-AS1 and miR-130a in different prognosis groups. (a) FGD5-AS1 expression levels in the GPG were markedly higher than those in the PPG (*t* = 5.205, *P* < 0.001). (b) miR-130a expression levels in the GPG were markedly lower than those in the PPG (*t* = 5.023, *P* < 0.001). (c) ROC curve; ∗∗∗ indicates *P* < 0.001.

**Table 1:** Primer sequence.

	Upstream primers	Downstream primers
FGD5-AS1	5′-GAAGGGCCGAAGAG CTCAAT-3′	5′-GGCTCGCAAAGTGTCTGTTG-3′
miR-130a	5′-GGCAGTCAATGCAATGTTAAAAG-3′	5′-CAGTGCGTGTCGTGGAGT-3′
GAPDH	5′-TATGATGATATCAAGAGGGT AGT-3′	5′-TGTATCCAAACTCATTGTCATAC-3′
U6	5′-CTCGCTTCGGCAGCACATATACTA-3′	5′-ACGAATTTGCGTGTCATCCTTGCG-3′

**Table 2:** Clinical data table.

	Observation group (OG) (*n* = 87)	Control group (CG) (*n* = 72)	*X* ^2^/*t*	*P*
Gender				
Male	39 (44.83)	41 (56.94)	2.314	0.128
Female	48 (55.17)	31 (43.06)		
Age (years)	48.1 ± 9.5	47.6 ± 8.5	0.346	0.730
BMI (kg/m^2^)	22.26 ± 2.46	21.75 ± 2.69	1.247	0.214
History of smoking				
Yes	39 (44.83)	23 (31.94)	2.749	0.097
No	48 (55.17)	49 (68.06)		
History of alcoholism				
Yes	18 (20.69)	11 (15.28)	0.774	0.379
No	69 (79.31)	61 (84.72)		
Number of teeth (teeth)	25.22 ± 4.05	26.57 ± 2.67	2.425	0.016
Gingival index	1.94 ± 0.58	0.21 ± 0.09	25.048	<0.001
Plaque index	1.43 ± 0.60	0.17 ± 0.06	17.736	<0.001
Sulcus bleeding index	2.63 ± 0.89	0.24 ± 0.11	22.632	<0.001
Pocket depth (mm)	3.93 ± 0.88	2.06 ± 0.47	16.213	<0.001
Attachment loss (mm)	4.22 ± 0.75	1.23 ± 0.27	32.134	<0.001

**Table 3:** ROC curve data.

Indicators	AUC	95% CI	Specificity	Sensitivity	Youden index	Cut-off
FGD5-AS1	0.835	0.769-0.901	88.51%	72.22%	42.21%	>0.805
miR-130a	0.851	0.792-0.910	80.46%	77.78%	58.24%	<1.227
Joint detection	0.929	0.891-0.933	80.46%	90.28%	70.74%	>0.321

**Table 4:** Univariate analysis table (*n* (%)).

	Good prognosis group (GPG) (*n* = 64)	Poor prognosis group (PPG) (*n* = 23)		
Gender				
Male	31 (48.44)	8 (34.78)	1.276	0.259
Female	33 (51.56)	15 (65.22)		
Age (years)	47.8 ± 9.9	49.0 ± 8.5	0.517	0.607
BMI (kg/m^2^)	22.45 ± 2.37	21.75 ± 2.69	1.172	0.245
History of smoking				
Yes	25 (39.06)	14 (60.87)	3.253	0.071
No	39 (60.94)	9 (39.13)		
History of alcoholism				
Yes	13 (20.31)	5 (21.74)	0.021	0.885
No	51 (79.69)	18 (78.26)		
Number of teeth (teeth)	25.33 ± 4.15	24.92 ± 3.80	0.415	0.674
Gingival index	1.84 ± 0.54	2.22 ± 0.60	2.811	0.006
Plaque index	1.31 ± 0.50	1.74 ± 0.75	3.075	0.003
Sulcus bleeding index	2.45 ± 0.87	3.13 ± 0.76	3.318	0.001
Pocket depth (mm)	3.73 ± 0.78	4.50 ± 0.88	3.924	<0.001
Attachment loss (mm)	4.25 ± 0.95	1.23 ± 0.43	5.547	<0.001
FGD5-AS1	0.59 ± 0.25	0.28 ± 0.23	5.205	<0.001
miR-130a	1.45 ± 0.41	1.93 ± 0.34	5.023	<0.001

**Table 5:** Assignment table.

Factor	Assignment
Gingival index	Data are a continuous variable and are analyzed using original data
Plaque index	Data are a continuous variable and are analyzed using original data
Sulcus bleeding index	Data are a continuous variable and are analyzed using original data
Pocket depth	Data are a continuous variable and are analyzed using original data
Attachment loss	Data are a continuous variable and are analyzed using original data
FGD5-AS1	Data are a continuous variable and are analyzed using original data
miR-130a	Data are a continuous variable and are analyzed using original data
Prognosis	Poor prognosis = 1, good prognosis = 0

**Table 6:** Multivariate analysis table.

Factor	*B*	S.E.	Wals	Sig.	Exp(*B*)	95% CI of Exp(*B*)	
						Lower limit	Upper limit
Periodontal pocket	1.398	0.694	4.054	0.044	4.047	1.038	15.782
Attachment loss	1.570	0.744	4.457	0.035	4.805	1.119	20.635
FGD5-AS1	-6.441	2.239	8.273	0.004	0.002	0.001	0.129
miR-130a	2.875	1.363	4.451	0.035	11.726	1.227	56.187

## Data Availability

The data used during the present study are available from the corresponding author upon reasonable request.
